# Efficient Multiuser Computation for Mobile-Edge Computing in IoT Application Using Optimization Algorithm

This article has been retracted.

**DOI:** 10.1155/2021/9014559

**Published:** 2021-11-10

**Authors:** Tawfiq Hasanin, Aisha Alsobhi, Adil Khadidos, Ayman Qahmash, Alaa Khadidos, Gabriel Ayodeji Ogunmola

**Affiliations:** ^1^Department of Information Systems, Faculty of Computing and Information Technology, King Abdulaziz University, Jeddah, Saudi Arabia; ^2^Department of Information Technology, Faculty of Computing and Information Technology, King Abdulaziz University, Jeddah, Saudi Arabia; ^3^Department of Information Systems, College of Computer Science, King Khalid University, Abha, Saudi Arabia; ^4^Faculty of Management, Sharda University, Uzbekistan

## Abstract

Mobile edge computing (MEC) is a paradigm novel computing that promises the dramatic effect of reduction in latency and consumption of energy by computation offloading intensive; these tasks to the edge clouds in proximity close to the smart mobile users. In this research, reduce the offloading and latency between the edge computing and multiusers under the environment IoT application in 5G using bald eagle search optimization algorithm. The deep learning approach may consume high computational complexity and more time. In an edge computing system, devices can offload their computation-intensive tasks to the edge servers to save energy and shorten their latency. The bald eagle algorithm (BES) is the advanced optimization algorithm that resembles the strategy of eagle hunting. The strategies are select, search, and swooping stages. Previously, the BES algorithm is used to consume the energy and distance; to improve the better energy and reduce the offloading latency in this research and some delays occur when devices increase causes demand for cloud data, it can be improved by offering ROS (resource) estimation. To enhance the BES algorithm that introduces the ROS estimation stage to select the better ROSs, an edge system, which offloads the most appropriate IoT subtasks to edge servers then the expected time of execution, got minimized. Based on multiuser offloading, we proposed a bald eagle search optimization algorithm that can effectively reduce the end-end time to get fast and near-optimal IoT devices. The latency is reduced from the cloud to the local; this can be overcome by using edge computing, and deep learning expects faster and better results from the network. This can be proposed by BES algorithm technique that is better than other conventional methods that are compared on results to minimize the offloading latency. Then, the simulation is done to show the efficiency and stability by reducing the offloading latency.

## 1. Introduction

The mobile application and Internet of Things (IoT) play a vital role and have placed a high demand on a wireless network and cloud infrastructure. The future of 5G communication is an important generation to the IoT because it needs the edge servers on a faster network with a higher quantity that can assist connectivity. The 5G spectrum expands the bandwidth frequency to transfer the data. The combination of edge computing and the next generation of cellular networks and computational networks from end-end devices can be offloaded accurately and on time by edge servers on base stations (BSs). To increase the communication and computation quantity of IoT systems, multiaccess edge computing (MEC) has recently developed the capable technology to solve this problem [1].

Edge computing for IoT has the aim to provide ecosystem capabilities for the IoT ROS-constrained by computation ROSs provided at the IoT network edge [2]. The multiuser-to-multiserver (MUMS) edge computing has a problem in ultradense cellular networks. The MUMS problem has been classified into two phases; they are server selection and offloading decision. In a single server environment, the users must register themselves to every application server; to overcome this issue, various methods of multiservers are developed. Nowadays, many scholars develop an open multiserver authentication scheme that can be proposed by using the literature of bilinear and ECC pairing [3].

The main goal is to exploit computational redundancy to reduce latency in a multi-user, multi-server network, by splitting the work generated by both sides into multiple works and offloading each work to a pool of mobile Edge Computing servers to a continuous execution that passes through the transmission Main channel [4]. The MEC concept was developed by the unparalleled growth of mobile traffic, specifically by smart mobile phones and the enhancement of multimedia services. Both multi-MEC and single-MEC server approaches consider the computation and communication limitations in the MEC environment [5].

The problem of allocating and freeing resources in the edge computing of mobile devices, where they do not have an account to calculate the allocation but must also have to allocate transmission to smartphone users through that account in the edge computing. Given a problem, they get decompose into task offloading issues; then, they solve using a heuristic approach and ROS allocation issues, which using the optimization techniques like convex and quasi-convex [6]. The Internet of Things (IoT) has some limitations like limited storage capacity, battery life is extending, or improving the application. These limitations are got decreased by improving the transmission of complex computations to devices, and the results are receiving from powerful devices like cloud, MCE, or fog; it is known as fog or edge-based method. Also, the smartphone devices and other objects have decreased the execution time, latency, and power savings using the offloading tasks on optimization techniques [7].

Offloading mechanism is based on the decision-making process; they have two types of strategies: static strategy and dynamic strategy; they depend on the time of offloading decision. The static offloading strategy is used for offline profiling that estimates the performance, and the dynamic offloading strategy performs the static analysis instrumentation and data to carry out the online profiling during execution time. However, IoT offloading is one of the most challenging topics, and they have more work to do in this area. IoT work can be accurate and speed to provide better performance with low latency for a wide range of IoT. The concept of IoT is used to collect the data from locally place sensor and pushed all the data from remote sensor and manipulate that into local device operations [8]. In which, the edge/fog computation is used to evaluate the real-world circumstances with IoT data to evaluate the benefits of providing fog and data offloading method in real-time that reduce the latency related to the design of cloud computing.

The number of network devices in the IoT ecosystem is constantly growing. The number of ROSs with the same service role is constantly expanding as well. ROS management is challenging due to the complexity of user needs. The selection of acceptable ROSs from among the many accessible ROSs to satisfy the expectations of users has become a top priority [9]. When compared to cloud computing, edge computing ROSs are limited when latency is reduced. Task scheduling, application performance, and user QoS are all affected by ROS availability and short-term forecasting. The ROS prediction technique can offer the appropriate ROS for customers by analyzing the ROS's load. As a result, in edge computing, predicting ROS QoS is critical for user experience and job allocation [10].

The new proposed optimization algorithm in metaheuristics is the bald eagle algorithm based on deep learning methods that are used, which is inspired by the real lifestyle of the bald eagles. There was intelligent in finding a place of fish hunting, them searching a place by keen observation, and then them swooping the fish at a well time. This The bald eagle algorithm has more living nodes, at the first stage they high in the number of living nodes but round increases the alive node decreases on an existing the system, [11]. By using this methodology in a limited time to predict a solution for a problem and it can be proven by nature-inspired computation in a better time, energy, living node analysis, and distance [12].

In the advent of the internet of things, the number of network devices increases, as in the demand on cloud data centers; some delay-sensitive service cannot be replied to in a timely manner, resulting in a decline in service quality (QoS) [13]. To address this issue, we offer a ROS estimation method based on QoS in edge computing in this research. To begin, the materials are categorized and matched based on their similarity in weighted Euclidean distance. Average rewarded is per time or per episode step that continuously taking action and observing the result that involves the continuous state and immediate reward. The matrix grey incidence is introducing for the matching function used for the ROS estimation method is done on BES select stage to reduce the offloading latency [14]. The suggested BES optimization model for mobile cloud computing (MEC) is based on a sensor that holds information on energy consumption, execution time, system dependability, and user experience quality (QoE). We have proposed an efficient offloading scheme that reduces the latency and time duration with energy-saving [15].

In this research, we follow an all-inclusive approach for task offloading with ROS allocation latency and scheduling with a special focus on delay on edge computing in IoT services. This can be encouraged by recent 5G technology on ultralow latency cases. Then, the latency and offloading can be optimized by using bald eagle optimization techniques. Hence, our contribution can be explained as follows:

- We mathematically defined and evaluate the bald eagle algorithm to reduce latency and offloading in edge computing as a BES algorithm
- Then explore the offloading and latency in IoT on 5G network in edge computing approach to efficiently solve the problem to optimality
- The numerical results show that the proposed task nearer offloading optimization algorithm provides a better achievement by using deep learning based on ROS estimation on edge computing between the consumption of power and task execution latency

The remaining sections that determine the offloading and latency between edge computing and multiusers under the IoT environment by new methodology are explained in this paper. Related work about mobile edge computing is explained in Section 2; system model is explained on Section 3; the main idea of the paper is explained in proposed methodology in Section 4; BES stages are explained in Section 5. Result and discussion of the research work to improve the efficiency are explained in Section 6, and the final part of conclusion for the research work has explained on Section 7.

## 2. Related Work

In maritime, users cannot happen the high requirement of transmission latency and power consumption; it causes due to the excessive traffic and limited ROSs in maritime networks [16]. To solve this problem, introduced a two-stage of the joint offloading optimal algorithm for maritime in mobile edge computing (MEC) is proposed; the two-stage of algorithms under the limited power and latency are optimizing computation and communication ROSs. They considered the latency dynamic tradeoff and consumption of energy. Offloading strategies and energy latency trade-offs are considering as the proposed methodology. In the future, they proposed the method to introduce by using artificial intelligence into the network in the ocean to explore the ocean and smart management.

Mobile edge has recently gained popularity. To improve the quality of experience, a potential paradigm has evolved for mobile devices from intense workloads computing growth (QoE). [17] presented the Gauss-Seidel and Lyapunov optimization methods, which are utilized to reduce the power consumption problem with task buffer stability, examine the specified trade-off and build an algorithm that offers local time complexity and offloading computation. MEC systems with several portable devices are often taken into account in this technique. The local execution mixed offloading computation techniques are obtaining combined design in which the mobile device tasks come at computing time in a stochastic way. The management of intelligent radio spectrum for offloading computing gets increasingly difficult as the number of devices grows (e.g., the transmit power). A performance analysis of the suggested algorithm was done, in which the trade-off between power consumption and computational efficiency delay effectiveness that can be avoided by utilizing this proposed technique was described clearly. For future investigation, many devices that might be relevant to the conclusions of this study should be considered.

[18] proposed a distributed computation offloading algorithm is Pt-based noncooperative game that achieve the Nash equilibrium. The numerical results that assess the mobile device impact on offloading decision-making users' behavioral biases. Mobile edge computing offers an effective solution for mobile devices with the delay task and computation intensive. To overcome the exciting problem of the mobile device is rational, and to maximize the expected objective utilities to make an offloading decision. By using the prospect theory (PT) to draw a framework, users formulate the decision-making of whether offload or noncooperative not as PT-based game [19]. Due to the uncertainty of the wireless channel and the less communication, the performance of computation offloading in MEC servers relies heavily on wireless access efficiency. They achieve the numerical results to analyze the impact of the biases of behavior on user's decision-making, and the multiple offloading users become smaller under the Pt-based model and then the classical EUT model

The problem detected are various splitting alternating direction methods of multipliers (ADMM), Gauss-seidel ADMM, Jacobi distributed ADMM and distributed improved Jacobi (DIJ)-ADMM algorithm they are solved by using proposed Alternating direction method of multipliers is applying on smart cities in that time [20]. The emerging applications on the smart cities are computation-intensive and time-sensitive; real-time vision processing applications are used in smart cities for their public safety and also in the virtual classroom. Both of the applications are hard to handle due to quick requirements of less time, and more computation is needed, to improve the development of smart cities by reducing the issues. Focus on task scheduling; it is critical issues to schedule a task for limited power, energy, and storage of mobile devices; to overcome these issues, by introducing these algorithms on the Internet of Vehicles (IoV) to handle and to reduce the optimization time and low cost are required; these are achieved by ADMM algorithm with fast convergence rate, and these four algorithms are better performance, and they reduce the task completion by increase the number of offloaded tasks [21].

[22] proposed the deep-Q network to reduce the computation offloading and ROS allocation. The requirement for Resource allocations for computation offloading through the Mobile Edge Computing (MEC); MEC provides the mobile stations to offload computation method to edge serve they positioned at the cellular network edge. To consider an efficient approach to relieve the computational burden and better computation offloading realize, the aim of the MEC is designed to joint task offloading and allocation of bandwidth with the low offloading cost, power cost, delay cost, and computation cost that every mobile station has number multiple methods that are being offloaded. The problem can be solved by using DQN techniques that can achieve near-optimal performance. The deep reinforcement minimizes the overall charges including the total consumption of energy and finishing the delay task. The method of DQN is better algorithm to evaluate the near-optimal solution. This proposed methodology is getting compared with MUMTO exciting algorithm [23].

To reduce latency and save energy can be computing nearby tasks of mobile users and enterprises in MEC system. The users make off-loading decisions, then the task to be considered. Offloading problems with NP-hardness, they are difficult in adapting to increase the dynamic and complexity of the application. To overcome these problems, [24] proposed a new methodology DRL-based offloading framework. They are automatically discovering the things from the various applications that infer an optimal offloading policy in different methods. This methodology shows that they better outperform the two heuristic baselines, and they achieve close optimal operation while having a complexity.

The multiaccess edge computing technology is used in 5G based on its capability to offload the computation workloads on mobile devices towards the edge approach to MD-specific limitations. Multitier multi-MEC activity is attracting interest in the 5G system. Two-tier computation offloading was explored as a method for MEC servers in the network, and it was necessary to assess the combined ROS allocation and computation offloading decision strategies in order to reduce the overall computational overhead of MD. The problem of allocating and freeing resources in the edge computing of mobile devices, where they do not have an account to calculate the allocation but must also have to allocate transmission to smartphone users through that account in the edge computing and reduce latency and save energy can be computing nearby tasks of mobile users and enterprises [25]. They developed the proposed method to resolve the difficulties of ROS allocation and computation trying to offload by particle swarm optimization, which is capable of producing high-quality solutions with guaranteed convergence. They outperformed several baseline methods on the optimization problem, reducing the total computing overhead of MDs. They are better at assessing the offloading optimization problem due to improved performance.

Mobile edge computing (MEC) is used to offload the computation tasks from user equipment's to the network edge to break ROS constraints and hardware limitations in 5G. [26] consider a small cell network planning to offload a task. To achieve energy efficiency, the consumption of an offload from both communication and task computation aspects. Scheduling of transmission is carried over both backhaul and front haul links. To solve the energy optimization problem, they develop an artificial fish swarm algorithm (AFSA). Various simulation results demonstrate the efficiency scheme.

The strategy is based on IoT device density and K-means algorithm to partition of network edge servers; then, algorithm is proposed for offloading decisions whether we need to offload the IoT devices; workload to edge servers and distribution of geographical various IoT devices can significantly improve the scheduling of network ROSs and satisfy the requirements [27]. The algorithm utilizing sample average approximation method is proposed to evaluate whether the tasks to be executed offloaded or locally. 20% of global cost is low than the benchmark on a true dataset of base station of Hangzhou.

[28] consider the offloading of sequential and parallel tasks on several MEC servers. They have been programmed to reduce the likelihood of failure as well as offloading delay. They presented an evolutionary algorithms and dispute graph models as two algorithms for solving the scheduling problem. This algorithm's performance, which was achieved by exhaustive search, shows that sequential offloading has a lower failure probability than parallel offloading that subtasks grow, and the latency gap among parallelized schemes narrows. [29] propose an energy-efficient deep learning-based offloading scheme (EEDOS) based on a smart decision-making algorithm that selects the best set of applications based on the user equipment's (UEs) remaining energy, supercomputing load, network conditions, communication delay, and data transfer amount. To reduce energy usage on UEs, offloading computation is performed on a nearby server.

## 3. System Model

Each base server is equipped with an edge server that has computing capacity that is limited. The transmission of data delay between the base server and edge server is so minimized. The distribution of geographical of users follows the geometric distribution. On the other side, each of the user devices generates a task of computing the Poisson distribution obeying in each time slot; then, the task of computing cannot be divided; the task must be processed either locally or offloaded.

The number of end devices and gateway can be considered on IoT networks. The number of end-devices and gateway can be considered in IoT networks is a director of The data from end-devices are getting collected by the gateway its coverage area and equipped edge server gets directly processes for that system.

The continuous various computation tasks are generated by the end device, and power and computation capacity are limited; the computation task may improve by offloading the tasks to the gateway in terms of task execution latency and consumption of power. The task offloading may focus on the representative of its own decision by end-end device making. The time horizon got discrete into epochs, duration *ƞ* equally with each epoch, and the multiple time epoch in time horizon is indexed by the integer 0 < *L* ≤ *L*; *L* is the multiple time epochs in time horizon each. The Fw represented as the frequency bandwidth, and the common license-free subgigahertz on end device operates the radio frequency.

The network in end devices is denoted as *T* = {*T*1, *T*2, ⋯, *Tn*} is a Network Representations. The assumed time varies between the end device and the gateway channel condition; the time slot *L* is the main channel condition.. The channel gain states are represented as *C* = {*c*^*k*^_1_, ⋯, *c*^*k*^_*n*_}. At each epoch time the channel condition, the *C* values are picked. The computation task of different independent by assuming every epoch to execute, they are indifferent sizes, and the CPU cycles are processed with different. The task queue is represented as *Q* = {*Q*_1_, ⋯, *Q*_max_} at the end devices, where *Q*_max_ is the multiple numbers of tasks stored at the end devices. Assumed that the task arrival as *P* = {0, 1}, where *P* = 1 that represents the generated task with its size that is randomly picked from *U* = {*u*_1_, *u*_2_, ⋯, *u*_*n*_}, otherwise, current time epoch no task arrived.

At the end device, the computation task can be executed, and the gateway got offloaded, and then at gateway got executed. At each IoT network, the computation task locally got executed by end devices, in the same time epoch the gateway got offload by their tasks. At first of the computation, each end device makes its own decision on offloading*K* = {1} ∪ {0} ∪ {−1}and the transmission power level*M*_*t*_ = {*M*^*k*^_1_, ⋯, *M*^*k*^_max_}to the edge devices; the offload end device is computed when*K*^*k*^ = 0; the local computation has cost only. Latency can be executed by the local and the power consumption; the power transmission is represented as *B*^*k*^_*t*_ = 0; in this cases *k*^*k*^ = 1 that represent the offload computation at the end devices to the gateway task, the transmission power *M*^*k*^_*t*_ *ϵ* *M*_*t*_. In some, both cases are executed successfully in computation task, and the outage between the end devices and gateway they suffer from the computational task, the execution of computation task fails, and *K*^*k*^ = {−1}.

The two different challenges in edge computing networks are the execution task latency and consumption of power; these depend on offloading scheme adopted task and transmission power allocation. We can evaluate the optimization problem to minimize the cost of the function by the consumption of power and execution latency.

The reachable edge servers for task offloading are needed to select by mobile users. The optimal offloading option obtain is an explosion combinatorial problem. In this research, a bald eagle search optimization technique is proposed to reduce the offloading latency in edge computing; the bald eagle algorithm (BES) is the advanced optimization algorithm that resembles the strategy of eagle hunting. The strategies are select, search, and swooping stages. Previously, the BES algorithm is used to consume the energy and distance; to improve the better energy and reduce the offloading latency in this research and some delays occur when devices increase causes demand for cloud data, the general idea of offloading strategy is explained in this flow chart process.

- First, according to the local strategy on grouping based on preferences, base servers are assigned by the mobile users with the high preference as the destination to offload tasks. The computation tradeoff of both distance and workload determines the preference. On one side, the base server and user are between closer distances; the preference value is larger. On another side, the base server's area is smaller workload; the preference value is larger
- The multiuser-to-single-server subproblem will be decomposed by the original problem, which means each base server is responsible for some users only. In individual groups, locally either process by local or task offloading. So, the selection problems 0-1 are subproblems; each subproblem is individually independent of each other; a distributed parallel can be processed
- Finally, the bald eagle search algorithm (BES) is used on the edge server by selecting, searching, and swooping stages that are working on BES algorithm to select the individually to end-end time to get fast and near-optimal IoT devices. They solve the problems 0-1 to get reduced the offload latency and get the near-optimal offloading decisions

The optimization objective is modeled as a very difficult 0-1 nonlinear optimization problem. On this problem, there is no polynomial-time complexity algorithm. Therefore, we are using a novel metaheuristic algorithm as a BES algorithm to reduce the complexity, and they used to obtain the approximate solution, and it is widely used in optimization problems.

### 3.1. BES Algorithm

The BES section introduces the major components of BES, which include the selection, scanning, and swooping steps. The remaining procedure is detailed, and to make BES implementation easier, Algorithm 1 provides the pseudo-code for the BES algorithm. The method was first triggered in Algorithm 1's first 1-2 lines. Initially, the Group O will produce in the problem situation, with the number of iterations *t* set to 0. The positional information is generated at random by each solution in O. After that, they assess each particle's goal. The following procedures are followed for each solution in subgroup O: The 4-12 lines use the best solution for looking about for picking an area, and the new area is assessed, as well as the searching and selection of regions using the spiral movement, which generates random numbers in two axes and two motions. By employing 13-21, the next point and the center point advance towards the answer, the seeking new location. Then, utilizing the swoop stage, the new position begins, in which the prey is searched for and swooped from the water. Use the solution lines in 22-30 to assess. In line 31, the iteration counter *j* is raised by 2. The previous evolutionary phase is repeated till the predetermined number of iterations is reached. Finally, the better solution achieved in the group is reported as that of the final rounds, and the solution in O is given as the final group.

### 3.2. Computation at Local Server

If *K*^*k*^ = 0, then the task of computation is done at the local end device. Let consider the edge server locates and the same CPU ROSs for each end device, and then, they executed at each time in the computation frame; assuming the time epoch *L*, *S*_*d*_ represents the multiple CPU cycles that required for 1-bit of input data in computation. CPU cycle that represents in per power consumption is *V*_*d*_. Then, the *S_d_V*_*d*_ represents the power consumption for computing per bit at the end devices. The one computation task in any epoch *L* at the end device then the total power consumption is denoted as *H*^*k*^_*cd*_, then is given by *H*^*k*^_*cd*_ = *S*_*d*_ *V*_*d*_MK. Moreover, let *y*_*d*_ denote the end device computation capacity; then, this measured by the number of CPU cycles per second. The remaining CPU ROSs are denoted by the remaining computation percentage ROSs *A*^*k*^ = {*a*_*d*1_, *a*_*d*2_, ⋯.1}. The latency of local computing *J*^*k*^_*d*_ is defined as *J*^*k*^_*d*_ = (*S*_*d*_ *m*^*k*^)/*Y*_*d*_. The two challenges are the consumption of power and the latency execution task in the edge computing network, simultaneously cannot reduce them by us; then, we try to achieve a better trade-off between them; then, the cost function is defined in the computation local server mode as

(1) $$\begin{array}{c} W_{loc}^{k}=H_{cd}^{k}+\alpha J_{d}^{k}, \end{array}$$

where *α* is denoted as the weight factor between the consumption of power and the latency of task execution.

### 3.3. Computing Offloading Load

Consider that the end devices that adopt the time division multiple access (TDMA) [30] are in multiuser method that transmit the data to the gateway, other end devices the interferences are negligible. When the data get transmitted over the equivalent time epoch, *R*, let *Q*^*k*^ denote the gain of the channel from any end device, during the offloading time epoch, is constant. *H*^*k*^_*t*_ indicates the power of transmission of the end device; then, the successful transmission rate (bit/s) is represented by

(2) $$\begin{array}{c} A_{k}=D_{w}\log_{2}\left(1+\frac{H_{t}^{k}Q^{k}}{\beta^{2}}\right), \end{array}$$

where *D*_*w*_ and *β*^2^ are represented as the bandwidth and the variance of additive white Gaussian noise (AWGN) individually. Then, the consumption of power on the end device that caused by the transmission of data as *H*^*k*^_*t*_ and the latency of transmission is represented as *T*^*k*^_*t*_ = *L*^*k*^/*A*_*k*_. Similarly, let *S*_*f*_ denote the frequency of computation at the edge server per CPU cycle. Let *f*_*s*_ indicates the capacity of computation located at the end devices. The power of computation is given by *C*^*k*^_*cs*_ = *S*_*f*_ *f*_*s*_ *m*^*k*^, and the latency computation is evaluated as *T*^*k*^_*s*_ = (*S*_*f*_ *M*^*k*^)/*f*_*s*_. Then, we can obtain the function of the cost of the computing offloading mode, and it is represented as

(3) $$\begin{array}{c} W_{\text{off}}^{k}=C_{cs}^{k}+H_{t}^{k}+\alpha \left(T_{s}^{k}+T_{t}^{k}\right). \end{array}$$

## 4. Proposed Methodology

### 4.1. Hunting Behavior of Bald Eagle

The name “Bald” comes from the ancient English word baldevgbyhuvu, meaning “White.” The bald eagles in this picture are not actually bald. Because of their size, they are sporadic predator and at the top of the food chain. They have been classified as scavengers since their food is readily accessible and high in protein. They mostly eat fish (living or dead), with salmon being their major source of nutrition. They determine that hinting is the best way to assess the energetic cost of a hunting endeavor; they use several attacking tactics to assess the calorific value of prey and their success in diverse environments. They love to hunt while flying and often from perches. They are capable of seeing fish from great distances, but catching one from the water is challenging. Only one of the attack's 20 tries was successful. They require recuperation after hunting since they use so much energy. They begin their quest for food by flying over the ocean. They begin by heading in a certain route and selecting a specific region for the food quest. Self-searching is used to locate available space, and they trail other birds for fish. The bald eagle's hunting activity is depicted.

Bald eagles will fly straight to the location. When compared to depth in the ocean, the success rate of the fishing eagle is higher at a radius of 5 km–6 km from the beach (47 percent–48 percent). The bald eagle's preferred habitat is the intermediate ground between the top and the water, where they choose their prey. A pair of eagles, in particular, is hunting together over 250 hectares of open grassland. Following the eagles' arrival over the region, they will begin their hunt; their selection area is no more than 650 m–700 m from their nest, since energy is a key component in searching.

While soaring in high, birds take advantage of the stormy weather. The rise in wind speed activates soaring, which causes the eagle to expend a significant amount of energy in order to fly. For hours at a time, they have been spotted flying gracefully, crawling, and unmoving. They have perfect vision, which allows them to see fish in the water or dead fish from hundreds of feet in the air. An eagle's eye is more potent and larger than a human's eye, and it has four times greater absolute vision. They can also see in two directions at once, side and forward vision perspectives. Eagles can fly over a hundred feet in the air, survey many areas at once with a twining motion, and detect prey from a distance of almost 2-3 meters.

An eagle's second stage of hunting is to locate prey; once they spot a fish, they go on to the last stage of hunting, which involves a steady flow of motion to reach a target at fast speed and capture it from the water. An eagle uses a consumption card that may estimate at branches of search power in the spiral when looking for prey.

## 5. BES Stages

This BES proposed an algorithm that imitates the behavior of bald eagle hunting skills that justify each stage of hunting. According to this Algorithm 2, they can be divided into three parts: the searching space for selecting, select from the select search space, and swooping the prey from the water.

### 5.1. Select Stage

In the select stage, the bald eagles are identified, and they select the best area within the search space select where they can hunt for fish. Equation (1) presents the behavior of hunting

(4) $$\begin{array}{c} O_{\text{new},\;}i=O_{\text{best}}+\beta *n\;\left(O_{\text{mean}}-O_{i}\right), \end{array}$$

where *β* is the parameter for controlling the position changes the values take between the 1.5 and 2 and *n* is a random number of the values between 0 and 1. In the selection stage, they are selecting an area based on information available from the earlier stage. They select random spaces that are different, but it is located near to the earlier search area. *O*_best_ denotes the search space that the eagle currently selected best position that is identified during the earlier search. In which, *O*_mean_ that indicates the eagle has used all the earlier point information. By multiplying the current movement of the bald eagle to randomly search prior information by *β*, they can randomly change all search points.

### 5.2. Search Stage

In this stage, bald eagles search for their prey from the selected space, and they move in a different direction than within a spiral space to hurry their search. The position for the swoop is expressed as

(5) $$\begin{array}{c} O_{i,\text{new}}=O_{i,\text{new}}=O_{i}+k\left(i\right)*\left(O_{i}-O_{i+1}\right)+l\left(i\right)*\left(O_{i}-O_{\text{mean}}\right)\\ k\left(i\right)=\frac{kn\left(i\right)}{\max\left(\left|kn\right|\right)},1\left(l\right)=\frac{\ln\left(i\right)}{\max\left(\left|lr\right|\right)}\left(1\right)\\ kn\left(i\right)=n\left(i\right)*\sin\left(\theta \left(i\right)\right),\ln\left(i\right)=n\left(i\right)*\cos\left(\theta \left(i\right)\right)\;\left(\text{ii}\right),\\ \theta \left(i\right)=b*\pi *\mathrm{rand}\cdots .\left(\text{iii}\right)\text{ and }n\left(i\right)=\theta \left(i\right)+N*\mathrm{rand}\;\left(\text{iv}\right) \end{array}$$

where *β* is a parameter of the values between 5 and 10 that determine the corner between the search point in the point of central and *N* takes the values between 0.5 and 2 to determine the cycle's search. The BES algorithm enables the new spaces and increases the diversification by multiplexing between the different current and next points of the polar in the *y*-axis. The *β* and *N* represent the parameter for change in a spiral shape.

### 5.3. Swooping Stage

In this stage, bald eagles get swing in the air from the search space their better position to target their prey. All points are move to the finest point. Equation (3) is represented as

(6) $$\begin{array}{c} O_{i,\text{new}}=\mathrm{rand}*O_{\text{best}}+u1\left(i\right)*\left(O_{i}-s1*O_{\text{mean}}\right)+v1\left(i\right)*\left(O_{i}-s2*O_{\text{best}}\right),\\ u1\left(i\right)=\frac{un\left(i\right)}{\max\left(\left|un\right|\right)},\;v1\left(i\right)=\frac{vn\left(i\right)}{\max\left(\;|\;vn\;|\;\right)},\\ un\left(i\right)=n\left(i\right)*\sin h\left[\theta \left(i\right)\right],\;vn\left(i\right)=n\left(i\right)*\cos h\left[\theta \left(i\right)\right],\\ \theta \left(i\right)=\beta *\pi *\mathrm{rand},\\ n\left(i\right)=\theta \left(i\right), \end{array}$$

where s1 and s2 ∈ [1, 2].

### 5.4. BES ROS Estimation Stage

We discuss about the ROS estimation function that relates with the same function. This is used for bald eagle function on their select stage to find the better ROS that reduces the latency to function it much faster. This estimation stage method consists of two phases such as similarity matching algorithm and the regression-Markov prediction chain method. Initially, we evaluate the matching degree of QoS ROS matrix between the user's requirement of QoS and the ROSs via similarity matching. This ROS matching satisfies the requirements of the users that are chosen by threshold. Finally, that we evaluate the changes of the load ROSs and the ROS optimal selection that can be done through the regression-Markov prediction chain method.

In edge nodes, the ROSs are provide to meet the requirement of QoS users. The set of ROSs that has a same function of service is defined as

(7) $$\begin{array}{c} P_{s}=\left\{p_{1},p_{2},\cdots \cdots p_{n}\right\}. \end{array}$$

The attributes of QoS that are requested by users are the same as ROSs. The attributes of QoS are represented as

(8) $$\begin{array}{c} aq=\left\{aq_{1},aq_{2},\cdots .aq_{m}\right\}. \end{array}$$

Each of the different ROSs on attributes of QoS, prediction technique can offer the appropriate ROS for customers by analyzing the ROS's load. According to the attributes, then the ROS is calculated to regulate the difference between the matching the user's needs and the ROSs. *Pq*_*i*_ as the ROS set that denotes the attributes of QoS group of ROS.

(9) $$\begin{array}{c} Pq_{i}=\left\{pq_{1},pq_{2}\cdots ..pq_{m}\right\}, \end{array}$$

where the *m* index that represent the ROS of each has different *m* on attributes of QoS that includes the availability, response time, price, and reliability. The attribute price is defined as

(10) $$\begin{array}{c} P=F*b\frac{\mu }{\varphi }*D_{{\text{dev}}^{\prime }}, \end{array}$$

where *F* is the service basic price, *μ* is the service number requests that is completed in per time, *φ* as the service number requests in per time, *b* as the adjustment price factor that can be determined by the provider service, and *D*_dev_ that represents the type of device that can be commonly divided into the small mobile devices, large mobile devices, and static devices. The ROSs of relative reserved in each device are in times, respectively.

The attributes of QoS are requested by the users that are the same as ROSs. The attribute of QoS is as follows:

(11) $$\begin{array}{c} aq_{i}=\left\{aq_{1},aq_{2}\cdots ..aq_{m}\right\}. \end{array}$$

To reduce the time matching and to improve the efficiency of matching, initially classify the ROSs before on the similarity matching, the attributes of QoS based on the requested values by the users, each of the ROSs is regarded in the point of the multidimensional space. Thus, the difference between the distance of the user needs and the ROSs is determined by the Euclidean distance.

The set of candidate ROSs satisfies the requirements of QoS users. Due to the uncertain nature and the dynamic of the ROSs, the value and amount of the information data on QoS collected will be fluctuate. The mobility inherent of the IoT makes the mobile users have volatility on certain using the ROSs. Therefore, we have a further ROS to select that the ROSs analyze the changes on load of the ROSs. Thus, the value of predictive is took into the state of corresponding interval to the solve of prediction value of interval. By using these basics, we can predict the ROS availability over a time period and select the right ROSs rationally.

To reduce the level of time matching and efficiency of matching, furthermore, ROSs are classified prior to matching similarity. On the basis of the QoS value requested by users, the multidimensional space can be considered as a point for each ROS. The distance between ROSs and requirement Euclidean distance is assessed by users. As every user may choose one attribute or every ROS attribute affects the measurement output differently, we set target weight per attribute and apply a weighted technique to calculate.

(12) $$\begin{array}{c} p\left(i,aq\right)=\sqrt{\overset{n}{\underset{i=1}{\sum }}g_{i}*{\left({fq}_{i}-{aq}_{i}\right)}^{2},}\\ p_{\text{sim}}\left(i,aq\right)=\frac{1}{1+p\left(i,aq\right)}, \end{array}$$

where *g*_*j*_ is a ROS attribute weight. The distance form *i*th ROS node *p*(*i*, *aq*) represents the spatial distance from the ideal node; this node refers to user's QoS requirements. The grade of nearness ranges between 0 and 1. *P*_sim_(*i*, *aq*) is smaller; the ROS is near the optimal node.

## 6. Simulation Performance

In this section, we determine the performance of the proposed offloading optimization techniques. The study of performance and behaviour of bald eagle hunting strategies and offloading optimization techniques proposed to reduce the offloading and latency between the edge computing and multi-users under the environments IoT. The existing methods were compared to get a better result. The important parameter on the performance includes the number of tasks, number of offloading power requirements, number of average rewarded task, and the latency requirement.

### 6.1. Experimental Results

Consider a multiuser in mobile edge computing (MEC) state in an IoT network. In this section, the IoT devices are randomly distributed within a 1 km area with edge servers in some heterogeneous. The IoT network is developing as one of the characteristics of core in 5G cellular network, which introduces a new environment coverage; there are many edge servers in the area of IoT devices. In this experimental result, there are many multiple users' choices of offloading end point for each user that can upload their tasks. Our proposed method goal is to achieve by assign all the tasks from different IoT devices to get most suitable edge servers to reduce the total latency.

That shows that the average power rewarded on per episode time interval tasks indexed different network scales in terms of edge servers. There is the number of users (user 1, user 2, user 3) using the network data from local to the edge computing, It can be incidental that the average reward achieved by BES algorithm; then, the solution is get improved, when it is compared to the existing method as DQN algorithm and DDPG algorithm.

That shows that the average task arrival rate of offloading latency on local in different user scales has a similar edge network. The number of users was developed and to reduce the offloading latency on edge computing data to the local. Average rewarded on task arrival rate decreases, while using edge computing by the local, it reduces the task arrival time.

That shows that execution of average power for the assigned task arrival rate per Mbps is compared with the BES algorithm that depends on edge computing; rewarded on per episode time interval tasks indexed different network scales in terms of edge servers the possible local area should serve the data and search by the nearer-edge computing network, which deals with more subtasks and have number of chances to avoid and reduce the power by using the edge serve on the task arrival rate.

That shows that the average latency and average buffering delays are measured in per ms between the distributed offloading on local are compared with BES algorithm is determined through the theoretical analysis on the figure. The task arrival rate of each task to the local on edge computing got delay latency, to attain the latency and buffering delay on between the local and the edge computing by using BES algorithm. It shows that we achieve the better results than the existing method. In this proposed method algorithm, used in this research work has more opportunities to continuous optimize the latency and offloading efficiency.

Researchers utilize the performance metrics as estimate indicators to test the performance of the estimate approach. The performance indicator as precision (prec = ∣*X* | /∣*Y*∣) is used to access the precision of ROS selection. Member ROSs that successfully match the user QoS account for a proportion of all ROSs. Recall (Rec = ∣*X* | /∣A ⋃ C∣). Specifically, the percentage of all matching successful ROSs is accounted for by the candidate ROSs that successfully match the user.

Figure 1 depicts the under varying matching criteria; there is a variation in accuracy and recall. Precision and recall are inversely related, as seen in Figure 2. The precision diminishes as the matching degree rises, but the recall increases. To ensure accuracy and recall within acceptable limits, the criterion *k* should be between 0.5 and 0.6. The change in *F*-measure under different matching thresholds is seen in Figure 2. The *F*-measure drops substantially as the threshold is raised. The *F*-measure is greater whenever the *K* value is 0.5; thus, *k* = 0.5 is selected as the matching criterion.

Figure 3 depicts the method's precision and recall performance, respectively. As we have shown, our technique regularly beats other techniques in term of accuracy, reaching 90%. Because the punishment factor enhances ROS similarity, it guarantees that ROSs are as close as feasible to the demands of consumers. The recall is, however, lower than for the other two approaches, remaining at 72 percent, also within acceptable limits. Although the technique is capable of ignoring restrictions and connections between ROS characteristics, it only matches the ROSs' quantity attribute and increases the prediction method's accuracy.

## 7. Conclusion

In this paper, we proposed a novel method as bald eagle search optimization technique to reduce the offloading and latency in mobile edge computing. The number of multiusers is used in IoT network to perform in better latency and to optimize the offload. We compare the BES algorithm with existing methods, by comparing the offloading, latency in number of multiusers at a computational time. Edge computing's local computation and storage capabilities can minimize latency and enhance user satisfaction. We employ weighted Euclidean distance similarity in this paper to classify several QoS attribute ROSs. By using similarity matching, we select the relevant ROS method. Finally, in order to balance user and service provider satisfactions and improve usage of ROSs, we can create a better approach for estimating ROSs. Experimental result indicates that the proposed system is an effective and shows the better results when it is compared with other two existing systems.

## Figures and Tables

**Figure 1:** Variation in precision and recall under different matching thresholds are used.

**Figure 2:** Variation of *F*-measure under different matching thresholds.

**Figure 3:** Similarity matching algorithm.

**Algorithm 1:** BES algorithm.

**Algorithm 2:** ROS matching.

## Data Availability

The data used to support the findings of this study are included within the article.
